# Relationship between Circulating BAFF Serum Levels with Proliferating Markers in Patients with Multiple Myeloma

**DOI:** 10.1155/2013/389579

**Published:** 2013-07-15

**Authors:** Michael G. Alexandrakis, Parascevi Roussou, Constantina A. Pappa, Ippokratis Messaritakis, Athina Xekalou, Nektaria Goulidaki, Anna Boula, George Tsirakis

**Affiliations:** ^1^Hematology Department, University Hospital of Heraklion, P.O. Box 1352, Stavrakia, 71110 Heraklion, Greece; ^2^Hematology Laboratory, University Hospital of Heraklion, Stavrakia, 71110 Heraklion, Greece; ^3^3rd Department of Internal Medicine, Medical School of Athens, Sotiria Hospital, 11527 Athens, Greece; ^4^Pathology Department, University Hospital of Heraklion, Stavrakia, 71110 Heraklion, Greece; ^5^Hematology Department, Venizelion Hospital of Heraklion, 71409 Heraklion, Greece

## Abstract

In multiple myeloma, there are many factors influencing the growth of the malignant clone in direct and indirect manners. BAFF is a growth factor for myeloma cells. The aim of the study was to measure its circulating levels in 54 pretreatment patients, along with serum levels of other proliferation markers, such as interleukins-6, -10, and -15, CRP, and beta-2 microglobulin, as well as bone marrow plasma cell infiltration and expression of Ki-67 PI, in various stages of the disease and after effective treatment in 28 of them. Serum levels of the previously mentioned factors were measured by ELISA, whereas bone marrow plasma cell infiltration and Ki-67 expression were estimated immunohistochemically. All measured parameters were higher in pretreated myeloma patients compared to healthy population and were also increasing with the progression of the disease. They all also decreased after effective therapy. Furthermore, all pretreatment values correlated to each other. BAFF seems to be an important growth factor for myeloma plasma cells. Measuring its serum levels, along with the previously mentioned cytokines, may provide important information regarding the degree of myeloma cells' proliferation. Therefore, they all could be used as markers of proliferation and disease activity.

## 1. Introduction

In multiple myeloma (MM) there is a malignant proliferation of monoclonal plasma cells, where multistep genetic and microenvironmental changes lead to the transformation of normal plasma cells into a malignant neoplasm. Progression events that can occur in all different molecular subtypes of MM include both genetic aberrations in MM cells (cytogenetic and epigenetic abnormalities, activating mutations of signaling pathways, and p53 deletion or mutation) and evolving interactions between different cell types within the BM microenvironment [1–3]. The adhesion of myeloma cells to hematopoietic and stromal cells induces the secretion of cytokines. 

Among them, interleukin-6 (IL-6) is a multifunctional cytokine involved in the pathogenesis of numerous diseases, including inflammation, autoimmunity, and lymphoid malignancies [4]. It is considered as the most relevant growth and survival factor for human MM. Its function as a survival factor is demonstrated by its ability to inhibit apoptosis induced by growth factor withdrawal, dexamethasone, and to trigger the expression of cell-death receptor Fas [5]. Interleukin-10 (IL-10), another cytokine, is probably the most potent inducer of immunoglobulin secretion by plasma cells in healthy individuals, together with IL-6 [6], being produced by numerous cell types, particularly normal and malignant B cells. IL-10 acts as a growth factor, in a paracrine and autocrine mode, for B cells, enhancing their proliferation, and moreover it is involved in their differentiation to plasma cells [6]. Elevated IL-10 levels have been detected in patients with MM, relating to the clinical status of the disease [7]. Interleukin-15 (IL-15) is a cytokine stimulating proliferation of cytotoxic T cells, regulating survival of NK cells and promoting proliferation and differentiation of preactivated B cells. In MM, it not only protects against spontaneous apoptosis but also against a broader range of death-inducing signals, including Fas-triggering [5, 8].

Ki-67 is a nuclear protein associated with cell proliferation. It has been used as a marker of proliferative activity in several human tumors, including MM. The monoclonal antibody to Ki-67 (MIB-1) is a marker strictly associated with cell proliferation, because it recognizes a nuclear antigen present during G_1_, S, G_2_, and M phases of the cycle, but not during the G_0_ phase. However, the determination of Ki-67 in MM is not a routine examination because there is little information regarding its clinical relevance and its association with prognostic factors [9, 10]. Ki-67 proliferation index (Ki-67-PI) represents the percentage of cells expressing the previously mentioned antigen and thus expresses the proliferation rate of the tissue.

B-cell activating factor (BAFF), also called B-lymphocyte stimulator (BLyS) and a proliferation-inducing ligand (APRIL) are TNF family members, critical for maintenance of normal B-cell development and homeostasis. Three receptors for BAFF have been identified: B-cell maturation antigen (BCMA), transmembrane activator, and CAML interactor (TACI) are common receptors for both ligands; BAFF-receptor (BAFF-R) is specific for BAFF, whereas heparan sulfate proteoglycanes, such as syndecan-1, are more specific for APRIL [11, 12]. The striking roles of BAFF and its receptors in normal B-cell homeostasis, as well as in several tumor models, raised the possibility that it may be involved in the pathogenesis of B-cell malignancies [13, 14]. It has been evident that myeloma cell lines and primary myeloma cells express BAFF and APRIL and their receptors, being both myeloma cell growth factors [15]. Addition of both ligands in MM cells may activate nuclear factor-kappaB, PI3K to Akt, and MAPK pathways and induces strong upregulation of Mcl-1 and Bcl-2 antiapoptotic proteins [16]. Furthermore, we have detected high serum BAFF levels in newly diagnosed MM patients, being correlated with disease stage and known factors of disease activity and decreased after effective treatment [17]. 

In the present study, we measured serum levels of BAFF in newly diagnosed MM patients in different stages of the disease and after effective conventional chemotherapy. Moreover, we correlated them with markers of myeloma activity, such as serum levels of IL-6, IL-10, IL-15, beta-2 microglobulin (B2M), and C-reactive protein (CRP), as well as with plasma cells' infiltration and Ki-67-PI in the bone marrow, both in diagnosis and after effective therapy.

## 2. Materials and Methods

### 2.1. Patients

We studied 54 newly diagnosed MM patients (28 male, 26 female, mean age 57 ± 14.5 years). According to the International Staging System (ISS), 16 were in stage I, 20 in stage II, and 18 in stage III of the disease. The paraprotein class was IgG in 29, IgA in 18, and light chain in 7 patients. Patients with liver or renal impairment, current or previous other malignancies or other bone marrow diseases, uncontrolled infectious diseases, use of immunomodulatory drugs, or incapability to consent were excluded from the study. None of the patients had received any kind of myeloma-related therapy prior to examination. We also studied 28 of them, after effective conventional chemotherapy, in complete or very good partial remission, when plateau phase was achieved. They had received the VCD (bortezomib, cyclophosphamide, and dexamethasone) (8 patients), Vel-Dex (bortezomib, dexamethasone) (7 patients), VMP (bortezomib, melphalan, and prednisone) (7 patients), and MPT (melphalan, prednisone, and thalidomide) (6 patients) regimens. As controls, 24 age- and sex-matched healthy volunteers were used. The work has been carried out in accordance with the Code of Ethics of the World Medical Association (Declaration of Helsinki) for experiments involving humans and according to the institutional review board guidelines and approved by ethical committee of the hospital. All subjects gave written and informed consent.

### 2.2. Measurements of Serum Concentrations

Serum samples were collected from patients and controls, aliquoted into separate vials, stored at −70°C, and assayed at the end of the study, in order to avoid interassay variability. Serum levels of BAFF, IL-6, IL-10, and IL-15 were measured using a commercially available sandwich enzyme linked immunoabsorbent assay (ELISA), employing monoclonal human anti-BAFF, IL-6, IL-10, and IL-15 (R&D Systems Inc., Minneapolis, MN, USA) according to the manufacturer's instructions.

### 2.3. Bone Marrow Examination

Both MM patients and controls underwent transiliac bone marrow biopsies being fixed in 10% formalin, decalcified in 10% EDTA and embedded in Paramat extra. Initially, haematoxylin and eosin stained, 3 *μ*m thick, sections were examined by light microscopy. The pattern and the percentage of bone marrow infiltration by myeloma plasma cells were highlighted by immunostaining them with a monoclonal antibody to CD38. Monoclonality and percentages of *κ*/*λ* neoplastic cells in the bone marrow were assessed by in situ hybridisation. 

After dewaxing and gradual rehydration, 3 *μ*m thick tissue sections were heated, cooled, blocked with 3% H_2_O_2_ in distilled water, and incubated with the primary monoclonal antibody anti-human Ki-67, (MIB-1 antibody, number M7240; Dako, Carpinteria, CA, USA) at a dilution of 1/50. At this point, blocking with H_2_O_2_ was repeated. After incubation with the Dako EnVision reagent/horseradish peroxidase conjugated polymer (kit 5007; Dako), the samples were exposed to diaminobenzidine tetrahydrochloride solution, washed with Tris buffered saline, and subsequently exposed to the second primary antibody (monoclonal anti-CD38, number M-7077; Dako), at a dilution of 1/50. The sections were then incubated with the EnVision reagent/alkaline phosphatase conjugated polymer (kit 1396; Dako), followed by incubation with the Fast Red chromogen plus levamisole. The sections were counterstained with Papanikolaou and Harris haematoxylin and coverslipped using glycergel aqueous mounting medium. Positive and negative controls were included in every run.

### 2.4. Statistical Analyses

Results are expressed as mean ± SD. The nonparametric Mann-Whitney test was applied to assess possible differences between untreated patients and control group. The nonparametric Kruskal-Wallis test and one-way analysis of variance (ANOVA) were assessed to test the existence of differences between different stages. Correlations between the various measured parameters were calculated by Spearman's rank correlation coefficient. *P* values <0.05 were considered to be statistically significant.

## 3. Results

Mean (±SD) serum levels for each of the analyzed parameters, as well as Ki-67 PI, in both patients and controls are shown in Table 1. All of them were found higher in MM patients compared to healthy population (*P* < 0.001 for all cases). Their values, according to ISS stage, are shown in Table 2. All of them had elevated values in parallel with disease progression (*P* < 0.004 for B2M and *P* < 0.001 for the other cases). Their values after effective treatment, in the phase of plateau, are shown in Table 3, where all of them decreased significantly compared to the pretreatment ones (*P* < 0.003 for CRP, *P* < 0.007 for B2M, and *P* < 0.001 for the other cases).

In the pretreatment group, serum levels of BAFF correlated positively with IL-6 (*r* = 0.711), IL-10 (*r* = 0.634), IL-15 (*r* = 0.642), Ki-67 PI (*r* = 0.693) (Figure 1), bone marrow infiltration (*r* = 0.530), and CRP (*r* = 0.330) (*P* < 0.02 for CRP, *P* < 0.001 for the other cases), and only a trend of correlation with B2M (*P* = 0.06) was noted. Similarly, IL-15 correlated significantly with IL-6 (*r* = 0.631), IL-10 (*r* = 0.664), B2M (*r* = 0.394), CRP (*r* = 0.357), bone marrow infiltration (*r* = 0.318), and Ki-67 PI (*r* = 0.631) (*P* < 0.02 for infiltration, *P* < 0.003 for B2M and CRP, and *P* < 0.001 for the other cases). Moreover, IL-10 correlated with IL-6 (*r* = 0.775), B2M (*r* = 0.273), CRP (*r* = 0.269), bone marrow infiltration (*r* = 0.369), and Ki-67 PI (*r* = 0.660) (*P* < 0.05 for B2m and CRP, *P* < 0.006 for infiltration, and *P* < 0.001 for the other cases). Ki-67 PI correlated with IL-6 (*r* = 0.775,  *P* < 0.001), B2M (*r* = 398,  *P* < 0.003), and bone marrow infiltration (*r* = 0.526,  *P* < 0.001); IL-6 correlated with bone marrow infiltration (*r* = 0.530,  *P* < 0.001), B2M (*r* = 0.455,  *P* < 0.001), and CRP (*r* = 0.271,  *P* < 0.05). Finally, B2M levels correlated with CRP (*r* = 0.339,  *P* < 0.01).

In the posttreatment group, values of IL-10 correlated with BAFF (*r* = 0.395,  *P* < 0.04) and IL-15 levels (*r* = 0.375,  *P* < 0.05), whereas only a trend for correlation was noted with IL-6 (*P* < 0.07). Furthermore, serum levels of B2M were correlated with B2M (*r* = 0.393,  *P* < 0.04).

## 4. Discussion

Recent studies support the notion that BAFF is essential for the survival of normal immature and mature B cells and normal plasmablasts. Dysfunctional BAFF signaling occurs in many B-cell neoplasias, with an autocrine loop stimulating the growth and survival of tumor cell [18]. BAFF plays an important role in the pathogenesis and propagation of MM due to its ability to promote B-cell survival, expansion, and differentiation. BAFF is present in MM cells and in the serum derived from patients with MM, suggesting an autocrine loop of stimulation from these tumor cells as well [15, 16]. Furthermore, osteoclasts seem to be among the predominant cell sources of both BAFF and APRIL, in bone marrow [19], suggesting that both ligands participate in the vicious cycle between myeloma cells and osteoclasts [20, 21]. In fact, it has been demonstrated that APRIL inhibition blocks partially the survival of MM cells supported by osteoclasts [21]. A positive correlation between BAFF expression and the activation of JNK pathway in human MM cells has been recently reported, suggesting that JNK activation and BAFF expression in MM cells may form a positive feedback loop promoting the survival and proliferation of MM cells [22] Moreover, activation of TACI receptor may upregulate *cyclin D2* and *integrin beta7*, following *c-maf* upregulation. This upregulation may promote malignant transformation of plasma cells through enhanced proliferation and adhesion with bone marrow stromal cells that can provide them survival signals [23]. It is of importance that neutralizing B-cell survival factors through binding to TACI receptor has shown clinical and biological activity in a phase-I study on MM and Waldenström macroglobulinemia [24]. In this study, we showed that BAFF levels are significantly higher in MM patients compared to healthy population. We also found that pretreatment BAFF levels differ significantly according to disease stage, since patients with advanced disease stage had significantly higher levels of BAFF compared to lower stages. This finding confirms previous observations indicating increased levels of BAFF in the serum of patients with MM [16, 17].

There are various factors correlating with MM progression. Among them, IL-6 is a potent myeloma cell growth factor, with both *in vitro* and *in vivo* activity. It is considered to be a significant prognostic marker in MM patients: not only is it higher in advanced stages or in progressive disease, in agreement with our results, but it also shows a strong correlation with several parameters of disease activity [7]. 

IL-10 exerts its biological functions primarily through STAT3. It has been recognized that IL-10 enhances the proliferation of B cells and promotes their differentiation into plasma cells [7, 25]. Moreover, it has been reported that BAFF induces IL-10-producing B cells in marginal zone regions, through activation of transcription factor AP-1 for binding to IL-10 promoter [26]. IL-10 has been involved in the activation of myeloma cells, supporting their long term growth responding to IL-6 [27]. Moreover, the concentrations of IL-10 in different clinical myeloma stages showed a positive correlation with disease progress [28]. We found elevated IL-10 serum levels in MM patients, compared to healthy population, as well as in advancing disease stage. Additionally, a significant correlation was noted between BAFF and IL-6 serum levels, suggesting the important role of IL-10 in myeloma progression.

IL-15, initially described as a T-cell growth factor [29], has been reported to costimulate the proliferation and differentiation of activated B cells [30]. IL-15 is expressed intracellularly by monocyte macrophages, dendritic cells, and fibroblasts [31]. IL-15 acts through a heterotrimeric receptor consisting of a specific high-affinity binding alpha-chain (IL-15Ralpha) plus the IL-2 receptor subunits beta- and common gamma-chain that mediate signalling [31]. IL-15 protects myeloma cells against spontaneous apoptosis [5]. An autocrine loop between IL-15 and its receptor has been identified as a mechanism for tumor cell expansion in MM [5]. The upregulation of IL-15 and IL-15Ralpha, in the B cells, suggests that this pathway is important in the pathogenesis for plasma cell tumors [7]. BAFF, as has been reported in the past, is able to mediate IL-15R upregulation [32, 33], whereas IL-15 may act synergistically with BAFF to B-cell growth. We demonstrated that serum IL-15 levels were elevated in MM patients and moreover in advanced disease, suggesting a crucial role in the mechanisms of B-cell proliferation and differentiation. Furthermore, we found correlations with BAFF, IL-6, and IL-10, suggesting that the previously mentioned cytokines are important mediators in the pathogenesis of MM.

Ki-67 is a nuclear protein being used as a proliferation index, since it is expressed only by dividing cells. In MM, it has been shown that it is correlated with markers of disease activity, whereas it may have prognostic value. Thus, Ki-67 PI > 8% has been accompanied with shorter survival [34], whereas values <4% are prognostic of better survival, independently from ISS [35]. Our results confirmed that Ki-67 PI correlated with ISS stage and disease activity and moreover with BAFF serum levels.

In this study, we found elevated serum levels of several growth factors, with differentiating potential, for myeloma cells in the newly diagnosed patients. All of them were increasing in advancing disease and subsequently decreased after effective treatment. Similarly, bone marrow infiltration and plasma cell Ki-67 PI, as direct proliferating markers, followed the same pattern. The decrease in the phase of plateau may be the result of the direct cytotoxic effect of the drugs on plasma cells, leading to a reduction in the release of cytokines from the myeloma cells, as well as to a reduction in their proliferation. Thus, serum levels of IL-6, IL-10, and IL-15 as well as bone marrow infiltration and plasma cell Ki-67 PI may be considered important indicators of disease activity. It is of importance that even in plateau phase, serum levels of IL-10 correlated positively with both BAFF and IL-15, which in turn correlated with B2M, suggesting their impact in the biology of the disease. The results of our study also link plasma cell proliferation to the cytokine milieu in MM patients, giving direct evidence for measuring their serum levels as proliferation markers.

More importantly, in the pretreatment group of patients, BAFF serum levels correlated significantly to all the aforementioned parameters of disease activity, whereas in the posttreatment group the correlation remained only for IL-10. This is in accordance with our previous study, which showed that BAFF levels correlated strongly with IL-6 as well as lactic dehydrogenase and C-reactive protein, which are also well-known markers of disease activity [17]. Our results support the fact that BAFF serum levels might have prognostic value.

## 5. Conclusion

Our results provide evidence that patients with active MM have raised BAFF, IL-6, IL-10, and IL-15 serum levels as well high Ki-67 expression of plasma cells in the bone marrow, whereas those of the posttreatment experience a significant reduction of these factors. All these parameters strongly correlate to one another. Thus, the assessment of serum levels of the studied cytokines as well as of the Ki-67 expression in bone marrow plasma cells may be considered proliferation markers and important indicators of disease activity. Further studies are needed in order to evaluate their possible use in future prognostic models.

## Figures and Tables

**Figure 1:** Positive correlations between serum levels of B-cell activating factor (BAFF) with interleukin-6 (IL-6) (a), IL-10 (b), IL-15 (c), and bone marrow plasma cell Ki-67 proliferation index (Ki-67 PI) (d) in multiple myeloma patients.

**Table 1:** Mean ± SD values of B-cell activating factor (BAFF), interleukin-6, -10, and -15 (IL-6, -10, and -15), C-reactive protein (CRP), beta-2 microglobulin (B2M), and Ki-67 proliferation index (Ki-67 PI) in multiple myeloma patients and controls (*P* < 0.001 in all cases).

	Controls	Patients
BAFF (pg/mL)	253.4 ± 171.9	904.2 ± 569.0
IL-6 (pg/mL)	1.0 ± 0.5	8.8 ± 7.8
IL-10 (pg/mL)	103.6 ± 16.8	170.4 ± 72.5
IL-15 (pg/mL)	5.6 ± 0.9	9.5 ± 4.7
CRR (mg/dL)	0.48 ± 0.23	1.02 ± 0.59
B2M (mg/L)	1.9 ± 0.56	3.75 ± 3.15
Ki-67 PI (%)	0.9 ± 0.9	9.3 ± 10.4

**Table 2:** Mean ± SD values of B-cell activating factor (BAFF), interleukin-6, -10, and -15 (IL-6, -10, and -15), C-reactive protein (CRP), beta-2 microglobulin (B2M), Ki-67 proliferation index (Ki-67 PI), and plasma cell infiltration among International Staging System multiple myeloma stages (*P* < 0.004 for B2M, *P* < 0.001 for the other cases).

	Stage I	Stage II	Stage III
BAFF (pg/mL)	498.5 ± 187.0	813.7 ± 398.3	1365.4 ± 641.5
IL-6 (pg/mL)	3.0 ± 1.2	6.2 ± 3.2	16.7 ± 8.5
IL-10 (pg/mL)	126.1 ± 26.0	150.3 ± 29.6	232.1 ± 91.9
IL-15 (pg/mL)	7.2 ± 1.2	7.7 ± 1.2	13.4 ± 6.4
CRR (mg/dL)	0.6 ± 0.3	0.9 ± 0.6	1.2 ± 0.7
B2M (mg/L)	1.8 ± 0.7	4.1 ± 3.5	7.4 ± 1.6
Ki-67 PI (%)	4.0 ± 2.4	7.1 ± 5.2	16.5 ± 14.6
Infiltration (%)	26.1 ± 10.8	39.4 ± 16.5	55.6 ± 14.6

**Table 3:** Mean ± SD values of B-cell activating factor (BAFF), interleukin-6, -10, and -15 (IL-6, -10, and -15), C-reactive protein (CRP), beta-2 microglobulin (B2M), Ki-67 proliferation index (Ki-67 PI), and plasma cell infiltration before and after effective treatment (*P* < 0.003 for CRP, *P* < 0.007 for B2M, and *P* < 0.001 for other cases).

	Pretreatment	Posttreatment
BAFF (pg/mL)	889.2 ± 681.4	303.4 ± 163.5
IL-6 (pg/mL)	7.5 ± 5.2	2.6 ± 1.3
IL-10 (pg/mL)	174.6 ± 77.0	131.3 ± 21.3
IL-15 (pg/mL)	9.5 ± 4.9	6.6 ± 1.8
CRR (mg/dL)	0.95 ± 0.66	0.51 ± 0.20
B2M (mg/L)	3.65 ± 3.19	2.06 ± 0.77
Ki-67 PI (%)	9.3 ± 7.5	2.7 ± 2.4
Infiltration (%)	39.4 ± 19.3	6.7 ± 5.1
